This article has been retracted.

# Cytokinin and abiotic stress tolerance -What has been accomplished and the way forward?

**DOI:** 10.3389/fgene.2022.943025

**Published:** 2022-08-09

**Authors:** Sayanti Mandal, Mimosa Ghorai, Uttpal Anand, Dipu Samanta, Nishi Kant, Tulika Mishra, Md. Habibur Rahman, Niraj Kumar Jha, Saurabh Kumar Jha, Milan Kumar Lal, Rahul Kumar Tiwari, Manoj Kumar, Radha, Dorairaj Arvind Prasanth, Abhijit Bhagwan Mane, Abilash Valsala Gopalakrishnan, Protha Biswas, Jarosław Proćków, Abhijit Dey

**Affiliations:** ^1^ Institute of Bioinformatics and Biotechnology, Savitribai Phule Pune University, Pune, Maharashtra, India; ^2^ Department of Life Sciences, Presidency University, Kolkata, West Bengal, India; ^3^ CytoGene Research & Development LLP, Barabanki, Uttar Pradesh, India; ^4^ Department of Botany, Dr. Kanailal Bhattacharyya College, Howrah, West Bengal, India; ^5^ School of Health and Allied Science, ARKA Jain University, Jamshedpur, Jharkhand, India; ^6^ Department of Botany, Deen Dayal Upadhyay Gorakhpur University, Gorakhpur, Uttar Pradesh, India; ^7^ Department of Global Medical Science, Wonju College of Medicine, Yonsei University, Wonju, Gangwon-do, South Korea; ^8^ Department of Biotechnology, School of Engineering and Technology, Sharda University, Greater Noida, Uttar Pradesh, India; ^9^ Department of Biotechnology Engineering and Food Technology, Chandigarh University, Mohali, India; ^10^ Department of Biotechnology, School of Applied and Life Sciences (SALS), Uttaranchal University, Dehradun, India; ^11^ Division of Crop Physiology, Biochemistry and Post Harvest Technology, ICAR-Central Potato Research Institute, Shimla, Himachal Pradesh, India; ^12^ Chemical and Biochemical Processing Division, ICAR-Central Institute for Research on Cotton Technology, Mumbai, Maharashtra, India; ^13^ School of Biological and Environmental Sciences, Shoolini University of Biotechnology and Management Sciences, Solan, Himachal Pradesh, India; ^14^ Department of Microbiology, School of Biosciences, Periyar University, Salem, Tamilnadu, India; ^15^ Department of Zoology, Dr. Patangrao Kadam Mahavidhyalaya (affiliated to Shivaji University Kolhapur), Ramanandnagar (Burli), Sangli, Maharashtra, India; ^16^ Department of Biomedical Sciences, School of Biosciences and Technology, Vellore Institute of Technology (VIT), Vellore, Tamil Nadu, India; ^17^ Department of Plant Biology, Institute of Environmental Biology, Wrocław University of Environmental and Life Sciences, Wrocław, Poland

**Keywords:** cytokinin (CK), CK metabolic genes, CK signaling genes, abiotic stress, crop resilience, genome editing

## Abstract

More than a half-century has passed since it was discovered that phytohormone cytokinin (CK) is essential to drive cytokinesis and proliferation in plant tissue culture. Thereafter, cytokinin has emerged as the primary regulator of the plant cell cycle and numerous developmental processes. Lately, a growing body of evidence suggests that cytokinin has a role in mitigating both abiotic and biotic stress. Cytokinin is essential to defend plants against excessive light exposure and a unique kind of abiotic stress generated by an altered photoperiod. Secondly, cytokinin also exhibits multi-stress resilience under changing environments. Furthermore, cytokinin homeostasis is also affected by several forms of stress. Therefore, the diverse roles of cytokinin in reaction to stress, as well as its interactions with other hormones, are discussed in detail. When it comes to agriculture, understanding the functioning processes of cytokinins under changing environmental conditions can assist in utilizing the phytohormone, to increase productivity. Through this review, we briefly describe the biological role of cytokinin in enhancing the performance of plants growth under abiotic challenges as well as the probable mechanisms underpinning cytokinin-induced stress tolerance. In addition, the article lays forth a strategy for using biotechnological tools to modify genes in the cytokinin pathway to engineer abiotic stress tolerance in plants. The information presented here will assist in better understanding the function of cytokinin in plants and their effective investigation in the cropping system.

## Challenging environmental factors and cytokinin

Climate change and rapid population growth pose enormous hurdles to achieving food security, which remains a primary concern for all stakeholders and governments (Muluneh, 2021; Dasgupta and Robinson, 2022). Feeding the rapidly expanding global population, which is anticipated to exceed 10 billion people by 2050 and needs 49% additional food, is a major challenge (Ahmar et al., 2020). There are already 820 million people in the world who are chronically undernourished, and this figure is expected to rise sharply in the future years, further compromising global food security (FAOSTAT, 2020). In addition, the hidden hunger is considerably worse today than it was a decade ago in Africa, Western Asia, and other developing nations (FAO et al., 2018). Furthermore, food production is being hampered by unusual weather circumstances connected to environmental degradation and rising land competition as a result of urbanization (Lobell and Gourdji, 2012; Lenaerts et al., 2019). Climate change is expected to raise the earth’s temperature, resulting in global warming, irregular rain patterns, and the intensification of various abiotic and biotic pressures, all of which significantly reduce agricultural yields (Raza et al., 2019). In the future, changing climate is expected to become more prevalent and aggravate different stress, posing major concerns to agricultural yield (Ray et al., 2013). In order to ensure sustainable agricultural production in the face of changing climatic and growing population, yearly crop yields must be increased (Tilman et al., 2011; Ray et al., 2013). Therefore, to address these multi-dimensional challenges, agricultural production systems must undergo a significant transition (Lenaerts et al., 2019). Sustainable agricultural production may be aided by the use of sustainable resources to boost crop yield per unit area and the effective usage of fertilizer and water. In order to alleviate the hidden and chronic hunger, economic development is essential, but it may not be sufficient to eradicate hunger (Lenaerts and Demont 2021). For thousands of years, plant breeding has been one of the most important strategies to fulfil people’s food needs *via* crop domestication (Ahmar et al., 2020).

Cytokinins are family of adenine-derived phytohormones characterised by the presence of an aromatic chain or isoprenoid at the N6 position of their adenine moiety (Mok and Mok, 2001). Cytokinins are typically defined as growth-promoting hormones, despite the fact that diverse substance with cytokinin action have been found to regulate wide range of developmental and physiological processes in plants. In the 1950s, Miller and Skoog identified the first cytokinin, kinetin, which was classified as a plant-derived molecule that accelerated cell division (Miller et al., 1956). A further investigation found that kinetin, in conjunction with auxin, was important for stimulating organ development and cell division in undifferentiated cells culture (Skoog and Miller, 1957). Despite the fact that the cytokinin study began in the mid-1900s, it is an ancient hormone, having emerged as one of the earliest hormones in photosynthetically competent organisms (Wang et al., 2015). According to evolutionary research, the genetic sequences that are orthologs to known components of the cytokinin signaling pathway may be found in the common ancestor of all land plants, charophytes (Wang et al., 2015). These findings indicate that cytokinin had a function in plants as far back as 450 million years. In addition, cytokinins are recognized for their role in plant growth, development, senescence delay, and modulation of biotic and abiotic stress tolerance (Kieber and Schaller, 2018; Cortleven et al., 2019).

Changes in chemoattractant, temperature, nutrient content, and osmotic conditions all activate cytokinin signaling cascades, which are evolutionarily connected to the two-component systems in unicellular organisms that engage in signal transduction (Hwang et al., 2002; Wolanin et al., 2002). Cytokinins perform critical and multifaceted functions in plant development and abiotic stress responses (Ha et al., 2012; Hwang et al., 2012; Zwack and Rashotte, 2015). Several research have shown that cytokinins have both positive and negative impacts on stress tolerance or resistance (Ghanem et al., 2008; Nishiyama et al., 2011). Plants, on the other hand, may experience both a short-term and long-term rise in cytokinin levels when they are exposed to extreme stress conditions (Alvarez et al., 2008; Dobra et al., 2010). For instance, cytokinin synthesis *IPT* genes (adenosine phosphate isopentenyl transferases) are up-regulated upon salt (NaCl) treatment, and a mutation in cytokinin biosynthesis leads to a robust salt-tolerant phenotype (Nishiyama et al., 2011). The impact of exogenous cytokinin administration on abiotic stress tolerance have been the subject of several investigations. *Triticum aestivum* (wheat) seedlings that receive exogenous cytokinins application are more tolerant to salt stress, whereas a similar treatment on *Phaseolus vulgaris* (beans) result in more susceptible phenotype to the salt stress (Kirkham et al., 1974; Abdullah and Ahmad, 1990). Furthermore, Arabidopsis plants displayed enhanced ability to survivie freezing or dehydration after being treated with endogenous cytokinin (Jones et al., 2010; Kang et al., 2012).

Transgenic plants that overexpress cytokinin biosynthesis genes (*IPTs*) or cytokinin degradation genes (*CKXs*) demonstrate the impact of altered endogenous cytokinin levels. More importantly, the overproduction of endogenous cytokinin enhances drought stress tolerance in many plants. However, reduced cytokinin levels, on the other hand, have a positive impact on drought tolerance (Werner et al., 2010; Qin et al., 2011; Macková et al., 2013; Li et al., 2021). Additionally, the cytokinin signaling components play a significant role in abiotic stress tolerance. For example, Arabidopsis *AHK1*, a histidine kinase 1 involved in cytokinin signaling, acts as a positive regulator of salt and drought stress responses. Furthermore, the loss-of-function mutant phenotype in *ahk2*, *ahk3*, and *ahk2 ahk3* in Arabidopsis is associated with increased tolerance to salt and drought stress (Wohlbach et al., 2008; Kumar et al., 2013). Drought stress responses are negatively and redundantly regulated by AHPs (histidine phosphotransfer proteins) (Hwang et al., 2012; Nishiyama et al., 2013). However, in salt stress resistance phenotype in Arabidopsis was discovered while researching the quadruple loss-of-function mutant *arr3arr4arr5arr6* (Mason et al., 2010). These early finding indicated that cytokinin metabolism and signaling genes play an important role in responding to diverse environmental stress conditions.

Cytokinin, on the other hand, cannot reduce abiotic stress on its own; instead, it functions in conjunction with other signaling pathways (Antoniadi et al., 2020; Li et al., 2021). There is a wealth of information available on the function of cytokinin and its interactions with other phytohormones when plants are exposed to abiotic stress. So, this review exemplifies the regulatory role of cytokinin in abiotic stress tolerance and activation of possible novel crosstalk with other key stress phytohormones. In this review, we provide an inclusive overview of the advancement of genetic approaches in dissecting the function of cytokinin signaling components in regulating stress tolerance in plants under challenging environments stress, followed by brief insights into future approaches.

## Plant mechanisms for sensing and response to abiotic stress

At the cellular level, several abiotic stressors such as drought, heat, cold, and salt may produce common cell disruptions and secondary stress such as membrane damage, reactive oxygen species (ROS) production and damage, protein denaturation, and osmotic stress (Figure 1). In general, the initial step in the stress response is perception, which is followed by the transmission of information through secondary messengers to regulators and, eventually, to effectors, which are responsible for the protective function. A sensor is a biological molecule that may detect an unfavourable change in its surrounding environment and immediately elicit a reaction by triggering the production of signal molecules inside the plant system. In general, receptors or membrane-associated proteins pick up on stresses, which causes an ionic imbalance across the membrane. Stresses caused by drought, heat, cold, and salt all induce an increase in the quantity of Ca^2+^ (signal molecules) that enters the cytoplasm of the cell from either its own reserves or an apoplastic source. One form of sensor for the stress signals is thought to be the passages that govern Ca^2+^ entrance (Aftab et al., 2021; Javaid et al., 2022; Paes de Melo et al., 2022). Other than Ca^2+^, ROS and nitric oxide (NO) are other messenger molecules involved in inducing plant response to cold stress. Plants generate ROS such as superoxide (O_2_), hydroxyl radicals (OH), and hydrogen peroxide (H_2_O_2_) in order to defend themselves against the diverse stress that they are exposed (He et al., 2018). In receptor-like kinases (RLKs), there is an extracellular domain, a transmembrane domain, and an intracellular kinase domain. The extracellular domain is where ligands bind, and the transmembrane domain is where protein-protein interactions take place (Ku et al., 2018). The histidine residue in the intracellular kinase domain is auto-phosphorylated when the ligand or signal binds to the extracellular domain, and the phosphoryl moiety is received by the aspartate receiver section of the sensor protein or a different protein (Yadav et al., 2021). After then, the activated sensor protein (or proteins) may either directly phosphorylate particular targets or trigger cellular responses that are unique to the signal that was received via the mitogen-activated protein kinase (MAPK) cascade. Protein phosphorylation and dephosphorylation, which are both forms of the intracellular signaling mode, govern a broad variety of cellular functions, including the activation of enzymes, assembly of macromolecules, localization of proteins, and their breakdown (Yadav et al., 2021). Plants are able to detect when they are being subjected to abiotic stress, which triggers a series of signaling cascades that activate ion channels, kinase cascades, the formation of ROS, and the accumulation of plant hormones, which ultimately leads to the induction of the expression of specific subsets of genes that are responsible combating the abiotic stress (Ku et al., 2018; Zandalinas et al., 2020). If the plant’s stress-coping systems are ineffective in reducing the negative consequences of stress, mostly due to ROS accumulation, the cells activate environmental-triggered cell death processes, which include the plant’s senescence (Zandalinas et al., 2020).

**FIGURE 1:** A simplified schematic representation of mechanism through which plant responses to diverse abiotic stress. The general signaling pathways in plants that are activated in response to abiotic stress, beginning with signal perception and leading to the stress responses. Cold, drought, light, nutrient and salinity frequently induce cellular damage and secondary osmotic and oxidative stress. Following upstream signaling processes and transcriptional controls activate stress-responsive mechanisms in order to restore cellular homeostasis and protect and repair damaged proteins and membranes after the initial stress signals (e.g., changes in temperature or osmotic and ionic effects or membrane fluidity). ABF, ABA responsive element (ABRE) binding factor; AP2/ERF, Apetala2/Ethylene Responsive Factor; bZIP, basic leucine zipper transcription factor; CAT, catalase; CBF/DREB, C-repeat-binding factor/dehydration-responsive-binding protein; CDPK, calcium-dependent protein kinase; COR, cold-responsive protein; HK1, histidine kinase-1; Hsp, heat-shock protein; ICE1, inducer of CBF expression 1; LEA, late embryogenesis abundant; MAP, mitogen-activated protein; PLD, phospholipase D; PX, peroxidase; ROS, reactive oxygen species; SOD, superoxide dismutase; and SP1, stable protein 1.

## Cytokinin in plant development and stress adaptation

Cytokinins are a family of plant hormones that are fundamental to a variety of growth and development processes (Pavlů et al., 2018). Cytokinins have been widely investigated for their metabolism, signal transduction pathway, chemical composition, and their role in plant growth and development, since their discovery in *Zea mays* (maize) seeds over 50 years ago (Figure 2). Inhibition of lateral root initiation, regulation of cell division, differentiation of metaxylem and phloem in roots, photomorphogenic cell differentiation in shoots and expanding leaves and inhibition or delaying of leaf senescence are all-important regulatory activity of cytokinins at the tissue and organ levels (Bielach et al., 2012; Chiang et al., 2012; Efroni et al., 2013; Zwack et al., 2015).

**FIGURE 2:** Cytokinin timeline: from discovery to crop plant application. A chronology of significant advancements in cytokinin research. Abbreviation: CKXs, CK oxidases/dehydrogenases; RRs, cytokinin response regulators; IPTs, isopentenyl transferases; HK, histidine kinas.

Adenine derivatives with aromatic side chains or isoprenoid make up the endogenous cytokinin. Isoprenoid cytokinin, which is abundant in nature, may be classified as trans-zeatin (tZ)-, isopentenyladenine (iP)-, cis-zeatin (cZ)-, or dihydrozeatin (DHZ)-type derivatives based on the side chain hydroxylation or reduction. In comparison, aromatic cytokinins, such as N6-(meta-hydroxybenzyl) adenine (BA), are less abundant in plants (Faiss et al., 1997). The isoprenoid cytokinins vary from one another in terms of their biological roles, metabolic conversions, biochemical characteristics, and transportability throughout the plant system (Pavlů et al., 2018). Cytokinin homeostasis is maintained by a number of enzymes engaged in cytokinin metabolism, including those involved in cytokinin production, inter-conversion between cytokinin types, and cytokinin degradation (Thu et al., 2017; Skalak et al., 2021). The role of a wide variety of genes and enzymes, along with the composed metabolic network controlled by cytokinins across the plant kingdom, has been thoroughly investigated (Zwack et al., 2015; Pavlů et al., 2018). The phospho-relay cascades of the two-component system (TCS) are established and lead to the expression regulation of specific genes involved in plant adaptation when the cytokinin signaling pathway is triggered by various environmental stimuli, like nutrition levels, changes in temperature, and osmotic conditions (Thu et al., 2017; Pavlů et al., 2018). Most recently, it was shown that cytokinin interacts with jasmonates (JAs), ethylene (ET), salicylic acid (SA), and abscisic acid (ABA), showing the presence of an interconnected coordinating network among the phytohormones involved in plant stress tolerance (Efroni et al., 2013; Thu et al., 2017; Artner and Benkova, 2019; Antoniadi et al., 2020; Skalak et al., 2021). Additionally, it is well established that cytokinin biosynthesis and signalling components operate as constitutive signals defining the plant response to drought stress and controlling drought acclimatization. Because of their spatiotemporal expression, rapid responses, and widely associated pathways, cytokinins are an ideal candidate for regulating complicated morphogenetic processes under water stress. We will highlight the importance of plant cytokinins and their regulation under abiotic stress in this review and will offer an approach to understanding the function and regulation of cytokinins in plants.

## Role of cytokinin in plant response and regulation to abiotic stress

Multiple aspects of plant growth and development are regulated by the phytohormone cytokinin. A significant number of mutants have been created in the cytokinin signaling pathway, biosynthesis, and breakdown processes, which has resulted in the rapid advancement in the field of cytokinin (Li et al., 2021; Prasad, 2022). According to research, cytokinins are important signaling molecules that trigger a range of plant stress responses. Moreover, abiotic stress has a direct effect on cytokinin transport, responses, and concentrations. Table 1 summarizes the genes from cytokinin pathways investigated so far that react to various abiotic stresses, in addition to their involvement in stress tolerance. We focused on nutrient, light, heat, drought, cold, and salt stress in this review to highlight the function of cytokinin in abiotic stress response and it is potential to increase abiotic stress tolerance (Figure 3).

**TABLE 1:** A summary of genetic research aimed at elucidating the function of cytokinin in the response to abiotic stress.

S. No	Plant species	Target genes	Expression under stress conditions	Genetic approach	Significant outcome	Reference
**Cytokinin biosynthesis**						
1	*Solanum lycopersicum*	*SlIPT3*	Strongly repressed in roots under salt stress	*35S:SlIPT3*	Improved tolerance to salinity	Žižková et al. (2015)
2	*Arabidopsis thaliana*	*IPT3*		*ipt3*		Žižková et al. (2015)
3	*S. lycopersicum*	*SlIPT4*	Strongly repressed in roots under salt stress			Žižková et al. (2015)
4	*A. thaliana*	*IPT8*		*ER:IPT8,* estradiol-inducible	Reduce plant tolerance under salt and osmotic stress	Wang et al. (2015)
5	*A. thaliana*	*IPT1*; *IPT3 IPT5*; *IPT7*		*ipt1 ipt3 ipt5 ipt7*	Increased resistance to salt stress, drought stress	Nishiyama et al. (2011)
6	*A. thaliana*	*CKX1*		*bGLU:CKX1 in barley*	Increased resistance to drought stress	Pospíšilová et al. (2016)
7	*O. sativa*	*OsCKX2*		*OsCKX2-RNAi*	Increased resistance to salinity stress	Joshi et al. (2017)
8	*O. sativa*	*OsLOG*	Downregulated by cold, drought and salt stress			Tripathi et al. (2012)
**Cytokinin homeostasis**						
9	*A. thaliana*	*UGT76C2*	Downregulated by osmotic stress and drought stresses	*35S:UGT76C2*	Tolerant to drought stress as adult plants	Li et al. (2015)
10	*A. thaliana*	*UGT76C2*		*ugt76c2*	More sensitive to drought stress	Li et al. (2015)
**Cytokinin signaling**						
11	*A. thaliana*	*AHK1*	Induced by dehydration	AHK1 overexpressor	Tolerant to drought stress	Liu et al. (2008)
12	*A. thaliana*	*AHK2*	Downregulated by salt			Buer et al. (2004)
13	*A. thaliana*	*AHK2*	Induced by dehydration	*ahk2*	Increased survival to drought after rewatering, increased survival upon salt stress	Liu et al., 2008; Argyros et al., 2008
14	*A. thaliana*	*AHK2*		*ahk2-2*	Hypersensitive to salt stress in terms of root growth and fresh weight	Zürcher et al. (2016)
15	*A. thaliana*	*AHK3*	Induced by hydration, high salinity and cold stress (3-week-old plants)	*ahk3*	Drought and salinity tolerant	Liu et al. (2008)
16	*A. thaliana*	*AHK3*	Not responsive to cold (11-day-old seedlings)	*ahk3*	Enhanced drought tolerance	Argyros et al., 2008; Tran et al., 2007
17	*A. thaliana*	*AHK3*		*ahk3-3*	Increased root elongation after transfer to low water potential media	Zürcher et al. (2016)
18	*A. thaliana*	*AHK2 AHK3*		*ahk2 ahk3*	More tolerant to drought and salt than single	Liu et al. (2008)
19	*A. thaliana*	*AHK2 AHK3*		*ahk2 ahk3*	Enhanced cold tolerance	Argyros et al. (2008)
		*AHK3 AHK4*		*ahk3 ahk4*		
20	*A. thaliana*	*AHK4*	Induced by dehydration			Liu et al. (2008)
21	*O. sativa*	*OsAHP1*		OsAHP-RNAi	Hypersensitive to salt treatment but resistant to osmotic stress	Jeon et al. (2013)
22	*A. thaliana*	*AHP2*	Downregulated by dehydration	*ahp2 ahp3 ahp5*	Strong drought-tolerant phenotype	Jeon et al. (2010)
23	*O. sativa*	*OsAHP2*		OsAHP-RNAi	Hypersensitive to salt treatment but resistant to osmotic stress	Jeon et al. (2013)
24	*A. thaliana*	*AHP3*	Downregulated by dehydration	*ahp2 ahp3 ahp5*	Strong drought-tolerant phenotype	Jeon et al. (2010)
25	*A. thaliana*	*AHP5*	Downregulated by dehydration	*ahp2 ahp3 ahp5*	Strong drought-tolerant phenotype	Jeon et al. (2013)
	*A. thaliana*			*ahp2 ahp3 ahp5*	Reduced type A *ARR* expression in response to cold	Sakai et al. (1998)
26	*A. thaliana*	*ARR1*		*35S:ARR1*	Hypersensitive cold response of type A *ARR*s as well as enhanced cold tolerance	Sakai et al. (1998)
27	*A. thaliana*	*ARR5*	Induced by cold, salinity and dehydration			Ha et al., 2013; Sakai et al., 2000
		*ARR6*				
28	*A. thaliana*	*ARR7*	Induced by cold, salinity and dehydration	*35S:ARR7*	Hypersensitive response to cold temperatures	Ha et al., 2013, Argyros et al., 2008
29	*A. thaliana*	*ARR9*	Weak and early induction by cold, downregulated by heat			Skalák et al., 2016; Ha et al., 2013
		*ARR10*				
30	*A. thaliana*	*ARR12*	Downregulated by heat stress	*arr1 arr12*	Less sensitive to salt stress	Skalák et al., 2016; Kang et al., 2013
31	*A. thaliana*	*ARR15*	Induced by cold, salinity and dehydration			Ha et al., 2013; Sakai et al., 2000
32	*A. thaliana*	*ARR22*	Weak and late induction by cold, induced by drought			Ha et al., 2013; Sakai et al., 2000
**Cytokinin response**						
33	*S. lycopersicum*	*SlCRF1*	Induced by cold in leaves and roots, repressed by heat in roots			Brenner et al. (2012)
34	*S. lycopersicum*	*SlCRF1*	Slightly reduced in leaves and strongly decreased in roots by drought			Brenner et al. (2012)
35	*S. lycopersicum*	*SlCRF2*	Induced by H_2_O_2_ treatment only in roots			Brenner et al. (2012)
36	*A. thaliana*	*CRF4*	Strongly induced in both root and shoot tissues by cold	*35S:CRF4*	Tolerant to cold treatment	Kang et al. (2012)
37	*A. thaliana*	*CRF4*		*crf4*	Sensitive to cold treatment	Kang et al. (2012)
38	*A. thaliana*	*CRF6*	Induced by heat shock, oxidative (H_2_O_2_) and salt stress			Reguera et al., 2013

**FIGURE 3:** Cytokinins function in plant development and abiotic stress. Schematic illustration of cytokinin as a signaling molecule that regulates key plant developmental processes and its response to various abiotic stress.

### Nutrient deficiency stress

Stress caused by nutrient deficiency in the soil triggers a number of reactions, all of which include cytokinin at varying levels (Pavlů et al., 2018). Root system architecture (RSA) is modified by the nutrients availability, and cytokinin is one of the important components that regulate RSA in response to availability of nutritional signals (Kroevoets et al., 2016). Nutritional signals affect the transcript levels of cytokinin metabolism and signaling genes, which are both implicated in regulating RSA (Bielach et al., 2012; Ramireddy et al., 2014; Chang et al., 2015; Pavlů et al., 2018). Cytokinin modulates the expression of various transporter genes as well as the development of passage cells, which affects the plant’s capacity to absorb nutrients (Werner et al., 2010; Andersen et al., 2018). As a result, cytokinin governs physiological and morphological adaptive responses to nutritional stress to survive. Furthermore, a study of the phosphate deprivation response in *Arabidopsis thaliana* mutants found that cytokinin signaling is essential for a significant response to decrease phosphate availability. This was the first study to demonstrate a specialized function for cytokinin signalling in nutritional sensing. (Franco-Zorrilla et al., 2002; Franco-Zorrilla, Martín et al., 2005). Sulfate transporter genes are suppressed by cytokinin, which is a negative regulator of sulphur acquisition (Maruyama-Nakashita et al., 2004). Cytokinin also inhibits genes involved in iron absorption and iron homeostasis (Séguéla et al., 2008). Cytokinin controls sodium (Na) build up through the sodium transporter gene *HKT1*;*1* as previously stated (Mason et al., 2010). Low potassium levels or an artificially reduced cytokinin status resulted in upregulation of the high-affinity K^+^ transporter gene *HAK5*, promotes root hair development, and accelerates ROS accumulation, indicating that cytokinin plays a role in responding to low potassium availability (Nam et al., 2012). However, another micronutrient, boron (B), was reported in *Brassica napus* seedlings to be linked to enhanced cytokinin content, which was thought to be a prerequisite for a different growth response (Eggert and von Wirén, 2017). Cytokinin is a key regulator in plant arsenic (As) stress adaptation (Mohan et al., 2016). Reduced cytokinin status was shown to make *A. thaliana* plants more resistant to arsenate, which is the most prevalent form of arsenic (As). Cytokinin deficit boosted the expression of As (V)/phosphate transporter genes and arsenate stress tolerance machinery, resulting in the aggregation of complexing agents (Mohan et al., 2016).

Higher cytokinin levels, on the other hand, induced tolerance to another soil pollutant, selenium (Se) (Lehotai et al., 2012). Subsequently these findings imply that cytokinin has a role in the regulation of As and Se stress adaption. Cytokinins capacity to regulate plant development in response to nutrient stress was demonstrated in recent research on the role of cytokinin in signaling the availability of nitrogen (N) from the roots to the shoots (Landrein et al., 2018; Poitout et al., 2018). The expression of a GFP reporter gene under the control of WUS promoter, that governs the expression of a key regulator of shoot apical meristem (SAM) activity, was measured using quantitative microscopy (Landrein et al., 2018). The analysis of reporter gene activation in the context of cytokinin metabolism mutants indicated that IPTs were necessary for *de novo* synthesizes of cytokinin in response to changed N supply in the soil. Increases in soil N content consistently enhances the concentration of tZR, which is the primary cytokinin transport form. The reaction of the *pWUS*:*:GFP* reporter gene to changing N availability happened quickly in the SAM, occurring within 24 h. Notably, grafting experiments between WT and cytokinin mutant plants demonstrated that while precursors to active cytokinins can be synthesized in the root (or elsewhere in the plant), the reporter gene response dependents solely on the ability of the shoot to form active cytokinins, presumably via LOG enzymes in the SAM (Chickarmane et al., 2012). Many studies have identified WUS as a primary target gene of RRBs (type-B response regulator proteins), suggesting a shorter signalling channel in the responsive meristem, which is consistent with cytokinin working *via* altering *WUS* activity (Dai et al., 2017). Poitout et al. (2018) determined that the ABCG14 transporter plays a critical role in the export of nitrate-induced cytokinin from roots, based on the fact that its mutation affected systemic N (nitrogen) signalling. Furthermore, they discovered a significant transcriptional reprogramming in shoots mediated by root-derived cytokinin, indicating that the hormone has functions beyond regulating SAM activity (Poitout et al., 2018). NLP transcription factors (TF), which act as positive regulators of *CYP735A* and *IPT* gene expression, are involved in the increase of cytokinin levels in the root in response to changes in nitrate availability. On the other hand, NIGT1 TF, which are also positively regulated by NLPs, act as negative regulators of *CYP735A* and *IPT* gene expression. (Maeda et al., 2018). The perennial grass *Lolium perenne* (Guo et al., 2017) produced results showing a role for cytokinin as a systemic N signal, implying that the function is evolutionarily conserved (Guo et al., 2017). Overall, it has been shown that cytokinin production in the root and translocation to the shoot contains significant information about soil conditions, particularly N availability, to the shoot, allowing the latter to control its own activity.

### Light stress

In addition to supplying energy for photosynthesis, light transmits information about the time of day and season, and it has an impact on the direction in which plants are growing. Excessive or insufficient light stress plants and new research indicates that an altered day/night cycle may also stress plants (Bhaskar et al., 2021; Li et al., 2021). The response to these pressures involves cytokinin at several levels, which will be briefly summarized in the sections that follows. Even though photosynthesis needs light, too much light can harm the photosynthetic apparatus as well as other parts of the cell. To prevent being stressed by too much light (high light stress), plants have evolved a number of defensive mechanisms, including the cyclic electron transport, disposal of excess light energy as heat, and light avoidance motions of chloroplasts and leaves (Takahashi and Badger, 2011). However, even with these protective mechanisms, exposure to excessive levels of light may induce an over reduction of the photosynthetic electron transport chain, resulting in photoinhibition, which reduces the efficiency of photosynthesis (Yamamoto, 2016). In particular, protein D1, which is a component of the reaction centre of photosystem II (PSII), is one of the most often affected by UV radiation (Edelman and Mattoo, 2008). Reduced cytokinin status resulted in lower photoprotection and increased photoinhibition in plants, owing to a significant fall in the D1 level (Cortleven et al., 2014). Additionally, due to inadequate D1 repair, cytokinin-deficient plants had a reduced ability to recover from photoinhibition after high light stress. Plants antioxidant capacity was also lowered as a result of a lack of cytokinin. Thus, multiple photoprotective systems were disrupted in cytokinin-deficient plants, demonstrating that the hormone is required for plants to survive under conditions of extreme light stress. *Arabidopsis histidine kinases 3* (*AHK3*) and, to a lesser degree, *AHK2*, and the type-B RRs, *Arabidopsis Response Regulators1* (*ARR1*) and *ARR12* were shown to be involved in the regulation of cytokinin activity (Cortleven et al., 2014). Additional evidence supports a protective role for cytokinin in the photosynthetic machinery under conditions of intense light (Cortleven and Schmülling, 2015). For example, cytokinin increases the antioxidant-based protection in chloroplasts, leading to an increase in the chloroplast’s lifespan (Procházková et al., 2008). Furthermore, because of the activation of the *PSARK*:*:IPT* gene, drought-stressed transgenic *N. tabacum* plants produced more CK and enhanced CO_2_ respiration, indicating that photosynthetic activities were well protected (Rivero et al., 2009). In comparison, another study reported that inhibiting cytokinin signaling in *A. thaliana* by mutating the *AHK2* and *AHK3* receptor genes showed an increased photooxidative stress tolerance under water deficiency circumstances (Danilova et al., 2014).

In addition, plants that have evolved unique response systems may be severely affected by a lack of light. In *A. thaliana* and *N. tabacum*, cytokinin is a key xylem-borne signal for photosynthetic adaptation to canopy light gradients (Boonman et al., 2009). Shade avoidance response is induced by low light, and it is characterized by the stimulation of elongation growth toward the light and the halt the growth of leaf in response. The shade-dependent auxin-induced degradation of cytokinin in developing leaf primordia is reliant on the *CKX6* gene, which has been discovered to be crucial. An increase in cytokinin degradation slowed leaf primordia development, saving resources for hypocotyl extension growth (Carabelli et al., 2007).

Light has the ability to transmit information about the time of day and to control the circadian clock. A prolonged light period has recently been revealed to generate stress symptoms in *A. thaliana* plants during the following night, a condition known as photoperiod stress (Nitschke et al., 2016; Nitschke et al., 2017). Plants suffering from cytokinin deficiency were the first to exhibit this phenotype, which could be described as following a standard sequence of events. An extended light period resulted in the induction of stress marker genes such as *BAP1* and *ZAT12*. Moreover, there is a significant increase in JA level several hours after the start of the night; the next day, a significant reduction in PSII maximum quantum efficiency (Fv/Fm) resulted in visible lesion formation in the leaves. When compared to cytokinin-deficient plants, WT plants displayed a considerably milder stress response, demonstrating that cytokinin plays a protective role. Cytokinin works primarily through *AHK3, ARR2*, *ARR10*, and *ARR12* and RRBs. After photoperiodic stress, several clock mutants (e.g., *cca1 lhy*) exhibited a significant stress response. Furthermore, stress sensitive clock mutants and cytokinin deficient plants shared a decreased expression or dysfunction of LHY and CCA1, two critical regulators of the circadian clock, indicating that a working clock is required to deal with photoperiod stress. Despite the fact that this novel kind of abiotic stress is ceased in natural settings, it is instructive regarding linkages between cytokinin and stress pathways that have hitherto gone unreported in the scientific community. It remains to be discovered what these “mechanical linkages” natural functions are.

### Cold stress

As a result of the membrane system hardening in low temperatures, cells become more vulnerable (Liu et al., 2016; Prerostova et al., 2021). Cold stress causes a number of physiological changes, including loss of membrane integrity, an imbalance between water and nutrients, and an increase in ion outflow. Cold stress triggers transcriptional and post-transcriptional regulatory processes that may be Abscisic acid (ABA) dependent or ABA independent (Prerostova et al., 2021). Low temperatures lead to the accumulation of ROS as the antioxidant enzyme activity is reduced which results in the failure of the proper functioning of the ROS scavenging system. As a result, an excessive accumulation of ROS will have harmful effects on the cell membrane, resulting in cell metabolism disorder and ion leakage (Sui, 2015). Additionally, low temperatures impair reproductive development. Cold stress during the flowering period of *O. sativa*, for example, will induce sterility and yield loss (Feng et al., 2014; Wang et al., 2017). Furthermore, when the temperature falls below 0°C, freezing stress develops, and the ice crystals formed leads to mechanical damage and metabolic dysfunction in plants (Liu et al., 2013; Cheng et al., 2014).

The effects of cold stress on energy generation and biochemical demand are profound (Koc et al., 2018). As a result, Zoysiagrass (*Zoysia japonica*) in high latitudes (relatively low-temperature regions) is more frost-resistant than Zoysia grass (*Z. japonica*) at low latitudes (relatively high-temperature areas). This might be because of the larger carbohydrate content employed as an energy store, as well as the involvement of phytohormones in controlling plant adaptation to cold temperatures (Li et al., 2018). *Carpobrotus edulis* produces more cytokinin under low-temperature stress, and an Arabidopsis mutant *amp1* with greater cytokinin concentrations displayed a higher relative growth rate and greater plant yield than WT (Xia et al., 2008; Khan et al., 2017; Fenollosa et al., 2018). Simultaneously, overexpression of *AtCOR15a*:*ipt* in *Saccharum officinarum* (sugarcane) increases cold tolerance by delaying leaf senescence and minimizing membrane damage, preventing significant production loss and freezing injury (Belintani et al., 2012).

Numerous studies have employed cytokinins to increase plant response to low-temperature stress. The multi-step phosphorylation mechanism is now the focus of research on the link between cytokinins and low-temperature resistance. According to some research, A-type *ARRs* such as *ARR5*, *ARR7*, and *ARR15* are positive regulators of *A. thaliana* cold tolerance (Shi et al., 2012). The C-type ARR *ARR22* contributes to low-temperature resistance in plants by keeping the membrane in a normal condition (Kang et al., 2013). When compared to the WT, B-type *arr1* mutant is more susceptible to low temperatures and has lower cold resistance, but *A. thaliana* with B-type ARR1 overexpression has higher cold resistance, suggesting that *ARR1* is a positive effector of cold signal transmission (Jeon et al., 2013). An *AHK2* or *AHK3* sends low-temperature signals to *ARR1* through *Arabidopsis histidine phosphotransfer proteins 2* (*AHP2*), *AHP3*, or *AHP5*, which shows that *AHP2*, *AHP3*, and *AHP5* plays an important function in upregulating tolerance to low-temperature stress (Jeon et al., 2013).

Plants low-temperature tolerance is further influenced by other cytokinin response factors (CRFs), which are discovered downstream of the cytokinin signaling cascade. Recent studies by Zwack et al. (2016) showed that *CRF4* is a positive regulator for the increased cold tolerance in *A. thaliana* with a *CRF4* mutation under low-temperature stress. An adaptation mechanism under cold stress may be triggered by high levels of *CRF2* and *CRF3* expression, which may stimulate lateral root development and overcomes the inhibition of cold-induced root growth, thereby increasing the plant’s ability to withstand low temperatures (Jeon et al., 2016). As a result, Arabidopsis with mutations in *AHK2*, *AHK3*, *AHK4* (cytokinin receptor histidine kinases) and *ARR7* (an A-type ARR) exhibits enhanced low-temperature tolerance, suggesting a function for these cytokinin receptor histidine kinases in cold stress signaling (Jeon et al., 2010). However, more experimental validation is required. Increased cytokinin levels, whether exogenous or endogenous, may enhance resilience to cold temperatures (Belintani et al., 2012; Jeon et al., 2016). Exogenous cytokinin pre-treatment may increase the cold tolerance of *Triticum aestivum* (wheat) seedlings exposed to cold stress by boosting endogenous cytokinin levels in the leaves (Veselova et al., 2005). Under cold stress, the administration of exogenous cytokinin in the *ahk* mutant is comparable to the higher-order mutation of AHK (a negative regulatory factor), which may increase plant cold tolerance. The molecular processes, on the other hand, remain a mystery Exogenous cytokinin treatment of wild-type plants has been shown to improve their ability to withstand cold stress. Furthermore, it has been claimed that certain A-type *ARRs* are positive regulators of the genes that control the response to cold stress. (Jeon et al., 2010). Type-A *ARRs* are extensively expressed in transgenic plants due to ARR protein stabilization (Shi et al., 2012).

When exposed to cold stress, the hormones ethylene (ETH) and cytokinin act antagonistically. The C-repeat binding factor/DRE binding factor (CBF/DREB) transcription regulation cascade is the most well-known cold signaling mechanism. An increase in cold sensitivity may be achieved by overexpressing CBF (Gilmour et al., 2000). ETH has been shown to negatively regulate the cold signal by regulating the expression of CBFs and A-type *ARRs* genes. Moreover, A-type ARRs are believed to be essential for integrating cytokinin and ethylene signals in regulating plant response to cold stress, and CBFs have been shown to negatively regulate the cold signal by modulating the expression of CBFs and A-type *ARRs* genes (Shi et al., 2012). The cytokinin signaling pathway or cytokinin-related transcription factors may be implicated in the response to cold, according to these studies.

### Heat stress

Heat stress damage the biological components by the production of ROS and proteins denaturation. It also has a detrimental impact on photosynthetic capability, resulting in a metabolic imbalance. The accumulation of heat shock proteins (HSP), which operate as molecular chaperones to prevent protein denaturation and aggregation, is one of the plant’s defence strategies against heat stress (Mittler et al., 2011). Heat stress decreases cytokinin levels, and exogenous cytokinin treatment usually improves heat stress resistance (Hare et al., 1997). In *Nicotiana tabacum* and *Agrostis stolonifera* (creeping bentgrass), for example, exogenous application of cytokinin and increased endogenous cytokinin concentrations reduced the inhibitory impact of heat stress on chloroplast and photosynthesis growth, increased antioxidant system activity, and upregulated heat shock proteins (Liu and Huang, 2002; Veerasamy et al., 2007; Xu et al., 2009; Xu et al., 2010). In *Oryza sativa*, *Zea mays*, and *Passiflora edulis* (passion fruit), cytokinin treatment improved thermotolerance of reproductive tissue and increase the yield of these plants, indicating that cytokinin is capable of priming heat stress defense (Sobol et al., 2014; Wu et al., 2016; Wu et al., 2017).

Photosynthetic capability is negatively impacted by heat stress, which affects chlorophyll concentration and photochemical efficiency (Fv/Fm) of leaves. Additionally, heat exposure increases ROS generation and protease activity, resulting in leaf senescence (Hu et al., 2020). Endogenous cytokinin levels in *A. thaliana* increase in response to heat stress, especially in the leaves, resulting in higher cytokinin concentration is essential for greater heat tolerance (Skalak et al., 2016). Furthermore, heat stress stimulates the generation of ROS, and higher cytokinin levels may activate the antioxidant system to eliminate ROS (Xu et al., 2009). Furthermore, hormone, proteome, and transcriptome study further reveal that cytokinin plays a critical role in plant tolerance to heat stress, with the majority of heat shock (HS) response proteins being elevated in response to higher cytokinin levels (Skalak et al., 2016). Under heat stress, however, when the cytokinin signaling pathway is disrupted and/or the concentration of endogenous cytokinin is decreased in Arabidopsis seedlings, the elongation of hypocotyls is significantly and continuously inhibited, both during the initial heat stress and during the subsequent seedling growth. The increase of endogenous cytokinins may preserve normal plant development under high-temperature stress and have a favourable effect on plants that have been treated with heat shock (Skalak et al., 2016). As a result, elevated levels of endogenous cytokinin may increase plant heat stress tolerance.

Introducing *isopentenyl transferase* (*IPT*) into *A. thaliana* seedlings boost endogenous cytokinin levels and hence increase tolerance to high temperatures (Skalak et al., 2016). As a result, boosting the amount of endogenous cytokinin in plants may help them to better withstand heat stress conditions. According to Skalak et al. (2016), the duration of elevated cytokinin levels is crucial for plant heat tolerance. The overexpression of the *IPT* gene under the start of continuous induction of expression promoters, such as the *HSP18* promoter or the senescence-activated promoter (*SAG12*), may be used to maintain high amounts of cytokinin. According to Xu et al. (2009), under heat stress, the overexpression of *SAG12*:*ipt* in *A. stolonifera* maintained the development and elongation of root systems, reduced chlorophyll loss and delayed leaf senescence, boosting plant heat tolerance. Subsequently, Xu et al. (2010) demonstrated that the overexpression of *IPT* generated by two separate promoters (*HSP18*:*ipt* and *SAG12*:*ipt*) results in a considerable increase in heat stress proteins in plants, boosting the plants ability to resist high temperatures (Xu et al., 2010). The DEX (dexamethasone) promoter (transient expression promoter)-driven overexpression of the *IPT* gene in *A. thaliana* may results in opening of stomata and leaf transpiration stimulation, both of which are important in the early stages of the heat stress response (Skalak et al., 2016). Furthermore, plant transpiration may only reduce the immediate demand for cooling, but it cannot alleviate the long-term impacts of heat stress because of its low water content (Wu et al., 2017). Increasing transpiration may only reduce the immediate requirement for cooling and cannot relieve the long-term impacts of heat stress owing to plants limited water content.

Along with boosting endogenous cytokinin content by *IPT* overexpression, a high level of cytokinin may be maintained by inhibiting endogenous cytokinin breakdown. Endogenous cytokinin breakdown may be inhibited in two ways. One of the methods is the mutation of the cytokinin oxidase/dehydrogenase (CKX) gene, while the other is through the use of cytokinin degradation inhibitors spray to decrease the activity of cytokinin oxidase/dehydrogenase (a negative regulator of cytokinin production). The CKX gene mutation causes an increase in cytokinin levels and grain production in *O. sativa*. Furthermore, in heat-sensitive *O. sativa* cultivars, CKX activity rises dramatically, resulting in poor cytokinin levels and yield. But the heat-resistant *O. sativa* CKX enzyme activity remains consistent, and the plants heat resistance improves (Wu et al., 2017). The CKX inhibitor INCYDE (cytokinin degradation inhibitor) is quite effective. The application of INCYDE boosts *A. thaliana* roots active cytokinin levels when exposed to heat stress (Zatloukal et al., 2008). On the other hand, Prerostova et al. (2020) have successfully demonstrated the opposite finding, that a single INCYDE treatment under heat stress had a detrimental influence on plant heat tolerance. The use of INCYDE in conjunction with acclimating plants may partially enhance *A. thaliana* heat resistance. Cytokinin response factors (CRFs) are thought to be a transcription factor that is linked to cytokinin. Under heat stress, *CRF1* expression in *Solanum lycopersicum* (tomato) roots is drastically reduced (Shi et al., 2014). Accordingly, we conclude that CRFs play a significant part in the plants heat stress signal pathway and that more study is required to elucidate the underlying process.

Moreover, exogenous cytokinin performs a similar effect to endogenous cytokinin when exposed to heat stress. Exogenous cytokinin zeatin ribose (ZR) treatment improves *A. stolonifera* heat tolerance by reducing root mortality, increasing the antioxidant system activity, maintaining a higher chlorophyll content, and upregulating related heat shock proteins (Veerasamy et al., 2007; Xu et al., 2010; Hu et al., 2020). To further boost plant growth and production, exogenous cytokinin has been implemented to enhance the heat stress tolerance of reproductive organs in plants.

### Salt stress

Salt stress affects numerous biochemical and physiological processes in plants. Accumulation of sodium ions (Na^+^) in plants may disrupt ion homeostasis, imbalance the potassium ion (K^+^)/Na^+^ ratio, and Na^+^ ion toxicity, all of which can result in secondary stress, including oxidative stress (Feng et al., 2015; Song et al., 2015; Liu et al., 2017; Guo et al., 2018). Moreover, ion leakage, cell membrane damage, and direct damage to proteins and other macromolecules are all caused by oxidative stress, which may result in cytotoxicity, membrane malfunction, and cell death in certain cases (Lin et al., 2018; Liu et al., 2018). Leaf senescence will be accelerated upon ion stress and oxidative stress, which will destroy the chlorophyll, limit photosynthesis and lower the yield (Han et al., 2011; Li et al., 2012; Liu et al., 2017). According to several research, the deleterious effects of salt stress on plants such as *Raphanus sativus* (radish) and *N. tabacum* are connected to cytokinins (Vankova et al., 2010). Under salinity stress, however, the alterations in endogenous cytokinins in various plants are not homogeneous. Due to the variability in cytokinin concentration under salt stress, there is no one-size-fits-all strategy for increasing plant salt tolerance via exogenous and endogenous cytokinin manipulation.

According to recent research, the cytokinin level of *Malus domestica* (apple) rootstock ‘robusta’ and *Solanum lycopersicum* seedlings remains high under salinity stress (Keshishian et al., 2018; Feng et al., 2019). Additionally, *A. thaliana*, *O. sativa*, and other plants exhibit an increase in cytokinin levels in response to salt stress (Prerostova et al., 2017; Joshi et al., 2018). The upregulation of cytokinin in certain plants may aid in the recovery from salt stress. Due to cytokinin accumulation, the *OsCKX2* knockout rice mutant exhibits a greater relative water content and yield under salinity stress than the WT, enhancing salt tolerance (Joshi et al., 2018). Moreover, increased plant resistance to salt stress may be achieved by increasing the activity of antioxidant enzymes by spraying INCYDE on S. lycopersicum. (Aremu et al., 2014). Avalbaev et al. (2016) showed that *Triticum aestivum* pre-treated with methyl jasmonate (MeJA) can maintain a high concentration of cytokinin by lowering the level of CKX transcription that is caused by salt stress, thereby delaying the negative impact of salt on seedling growth, and enhance salt resistance (Avalbaev et al., 2016). In response to the deletion of 42 bp from the promoter region of *IPT5* gene, the expression level and cytokinin content of *M. domestica* rootstock “robusta” under salinaty stress were both increased, with the latter remaining at a high level and exhibiting greater tolerance to salt stress (Feng et al., 2019). *SlIPT3* overexpression makes *S. lycopersicum* more salt-tolerant by keeping their photosynthetic pigment and K^+^/Na^+^ ratio high, which means they can withstand more salt than the WT plants (Ghanem et al., 2011).

High cytokinin concentration, on the other hand, have been demonstrated in experiments to reduce plant salinity tolerance. Furthermore, overexpression of *AtIPT8* in *A. thaliana*, which has a high cytokinin level, results in a substantial reduction in the survival rate of plants under salt stress. This is due to the downregulation of stress-responsive genes, the inhibition of the antioxidant system, and the reduction of chlorophyll content in the plants (Wang et al., 2015). Furthermore, plants with lower cytokinin levels have been reported to be more resistant to abiotic challenges, such as salt stress, owing to decreased cytokinin production or increase degradation (Ghanem et al., 2011; Avalbaev et al., 2016; Zhang et al., 2018). In comparison to the wild type, salt tolerance is higher in cytokinin synthesis pathway mutants with loss-of-function mutations, such as *Atipt1*, *Atipt3*, *Atip5*, and *Atipt7* (Nishiyama et al., 2012; Zhang et al., 2018). In the moss *Physcomitrella patens*, overexpression of *PpCKX1* lowers cytokinin levels and increases salt tolerance (Hyoung et al., 2019). Salt tolerance in transgenic *Medicago sativa* (alfalfa) plants is improved by overexpression of *MsCKX*, which maintains a high K^+^/Na^+^ ratio and increases the activity of antioxidant enzymes to scavenge ROS (Li et al., 2019). These CKX-induced cytokinin-deficient plants are more valuable for deciphering the function of cytokinin than *ipt* mutants (Werner et al., 2003).

Plant salt tolerance is also influenced by components in the cytokinin signaling system. The cytokinin receptor *AHK1* is a positive regulator of salt stress response and plays an active regulatory function in osmotic stress signaling (Tran et al., 2007). Furthermore, plant tolerance to salt is improved by *ahk2*, *ahk3*, and *cre1* mutants, which upregulate the expression of homologous stress response genes, indicating that these members have a negative regulatory function in salt tolerance (Tran et al., 2007). By promoting the expression of *A. thaliana high-affinity K* ^*+*^ *transporter 1;1* (*AtHKT1;1*) in the roots, the *arr1* and *arr12* mutants decrease sodium accumulation in the aerial portions and improve salinity stress tolerance (Mason et al., 2010). Overexpression of *ARGONAUTE2* (*AGO2*) in *O. sativa* decreased cytokinin concentration in shoots and increase cytokinin level in roots, resulting in higher salt tolerance and grain length in *O. sativa* under salt stress, according to Yin et al. (2020). In addition, by boosting the production of *BIG3* (*GRAIN3*), which encodes a protein that may be involved in cytokinin transport, and AGO2, which changes the histone methylation level of BG3, AGO2 impacts the distribution of cytokinin. CRFs are thought to be downstream signaling molecules for RRs in certain instances (Hallmark et al., 2019). Consequently, under salt stress, RNAi silencing of *ThCRF1* reduced salt tolerance in *Tamarix chinensis* (halophyte: salt-tolerant plants), while overexpression of *ThCRF1* greatly increased salt tolerance in the halophyte through regulating osmotic potential and increasing antioxidant enzyme activity (Qin et al., 2017).

Depending on the plant species and the degree and duration of salt stress, increase or downregulation of cytokinin improves salt tolerance. Exogenous cytokinin treatment has a range of impacts on tolerance of salt stress in plants of different species. Although pre-treatment of legumes with exogenous cytokinins increases their susceptibility to salt, most research has shown that exogenous cytokinins improve plant salt tolerance, particularly in cereal crops like *O. sativa* and *T. aestivum* (Iqbal et al., 2006; Javid et al., 2011). By efficiently relieving salt-induced leaf senescence and other forms of physiological or developmental damage, foliar application of 6-Benzylaminopurine (6-BA; synthetic cytokinin) improves *Solanum melongena* (eggplant) and *Lolium perenne* (perennial ryegrass) salt resistance (Wu et al., 2014; Ma et al., 2016). These findings suggested that we can spray exogenous cytokinins onto plants to improve salt resistance.

### Drought stress

Reduced photosynthesis, decreased crop yields, and accelerated senescence is some of the negative consequences that drought stress may have on plant physiological activities (Liu et al., 2012; Zheng et al., 2017; Hai et al., 2020). Subsequently to salt stress, the likelihood of increasing plant drought resistance via cytokinin regulation is dependent on the stress duration, plant dehydration rate and soil water potential, (Veselov et al., 2017). Furthermore, endogenous cytokinin upregulation and downregulation have both been reported to increase drought tolerance. (Werner et al., 2010; Zhang et al., 2018). According to several research, under drought stress, plant endogenous cytokinins accumulation is decreased, and this leads to improving plant drought tolerance through a variety of physiological responses such as early leaf senescence, leaf abscission and stomatal closure (Xu et al., 2016; Naidoo and Naidoo 2018; Calvo-Polanco et al., 2019). Moreover, cytokinin is a negative regulator of plant root development and branching, enhancing cytokinin breakdown in the root may result in plants with an improved root-to-shoot ratio, larger root system, and long-term drought resistance (Pospisilova et al., 2016; Ramireddy et al., 2018).

Overexpression of CKX causes cytokinin to be downregulated, resulting in slower plant development and higher protective chemical content (proline, betaine, etc.) as well as drought resistance in *A. thaliana*, *N. tabacum*, *Cicer arietinum* (chickpea), and *Hordeum vulgare* (barley) (Werner et al., 2010; Nishiyama et al., 2011; Pospisilova et al., 2016; Ramireddy et al., 2018; Khandal et al., 2020). In *A. thaliana*, the *ipt1*, *3*, *5*, and *7* mutants had lower endogenous cytokinin content and improved drought tolerance (Nishiyama et al., 2011). Reduced levels of cytokinin cause roots to expand and shoot to have a higher root-to-shoot ratio, which improves root surface area available for water absorption. Smaller branches and leaf areas in comparison to roots may significantly reduce transpiration which further improves the tolerance (Werner et al., 2010; Lubovská et al., 2014; Prerostova et al., 2018). Accordingly, the whole plant can keep a relatively high relative water content and become more drought-resistant. Furthermore, by counteracting the effects of the oxidase system, downregulation of cytokinin may contribute to an improvement in drought tolerance (Lubovská et al., 2014). Conventional multi-step phosphorylation system in plants, including RRs, HKs, and HPs, is responsible for cytokinin signaling in the plant. Cytokinin signaling is also regarded to be a negative regulator of drought resistance because *ahk2*, *3*, *5*, *arr1*, *10*, and *12* display a significant drought-tolerance phenotype (Kang et al., 2012; Nguyen et al., 2016). Since the cytokinin signal suppresses stress response gene expression, it is hypothesized that decreasing the amount of cytokinin in the plant might enhance plant survival under challenging environmental conditions (Zhang et al., 2018). Moreover, it was shown that the expression of *SlCRF1*, *SlCRF2*, *SlCRF3*, and *SlCRF5* was regulated throughout the drought and recovery phase in *Solanum lycopersicum* plants, demonstrating that CRFs respond to drought stress and providing a novel idea for improving plant resistance to drought stress (Gupta et al., 2014; Shi et al., 2014).

Drought, salt, and cold stress all results in reduce water availability, resulting in physiological reactions that overlap. Different strategies have been developed in plants to optimize the use of water, including redirection of root development, change of cell membrane characteristics, and control of transpiration via stomata (Feng et al., 2016; Zhu, 2016). Moreover, drought response is tightly linked to the activity of abscisic acid (ABA), which increases in response to drought stress and binds to its corresponding receptor family PYRABACTIN RESISTANCE1 (PYR1)/PYR1LIKE (PYL)/ABA RECEPTOR REGULATORY COMPONENTS (RCAR). An enzyme called PROTEIN PHOSPHATASES 2C (PP2c) is inhibited by the ABA-PYR/PYL complex. When ABA is absent PP2c dephosphorylate and keeps subclass III SUCROSE NONFERMENTING1 (SNF1)–RELATED PROTEIN KINASES2 (SnRK2s) inactive. Furthermore, SnRK2s that have been activated phosphorylate transcription factors known as ABRE BINDING FACTOR (ABFs)/ABSCISIC ACIDRESPONSIVE ELEMENT (ABRE) BINDING PROTEINS (AREBs), which control the expression of target genes to promote plant drought tolerance (Miyakawa et al., 2013; Joshi et al., 2016). Moreover, drought and osmotic stress activate another signaling pathway that is independent of ABA and includes GROWTH REGULATING FACTOR7 (Kim et al., 2012).

Drought reduces cytokinin levels in *A. thaliana* and *Glycine max* (soybean) by repressing *IPT* genes and upregulating *CKX* genes (Guo and Gan, 2011; Nishiyama et al., 2011; Le et al., 2012; Nishiyama et al., 2013; Ramireddy et al., 2014; Nguyen et al., 2016; Todaka et al., 2017). Moreover, genetic studies in *A. thaliana* have consistently shown that cytokinin functions as a negative regulator of drought stress tolerance, which is consistent with previous findings (Nishiyama et al., 2011; Nishiyama et al., 2013; Nguyen et al., 2016). Furthermore, lowered cytokinin levels and signaling resulted in at least two primary effects: greater sensitivity to ABA, establishing cytokinin as an ABA antagonist and a decrease in shoot growth, which is an adaptive response to drought (Werner et al., 2003; Riefler et al., 2006). Numerous components of the cytokinin signalling that are functionally significant in the tolerance to drought stress have been established (Li et al., 2016). Therefore, plants with mutant cytokinin receptor genes (*AHK2* and *AHK3*), HPT genes (*AHP2*, *AHP3*, and *AHP5*), or RRB genes (*ARR1*, *ARR10*, and *ARR12*) exhibited greater drought stress tolerance compared to control plants (Nishiyama et al., 2011; Nguyen et al., 2016). However, drought tolerance was connected with a variety of physiological changes, including an increase in cell membrane integrity, reduction in stomatal aperture, and an increase in ABA sensitivity (Nguyen et al., 2016). According to a transcriptomic study, cytokinin regulates a large number of dehydration/drought and/or ABA-responsive genes involved in drought adaptation (Nguyen et al., 2016). Increasing evidence suggests that under drought and salt stress, the RRA genes *ARR5*, *ARR6*, *ARR7*, *ARR15*, and *ARR22*, which also react to cold stress in a cytokinin independent manner, were upregulated, showing a partial overlap of the response pathways (Kang et al., 2012; Jeon and Kim, 2013). Drought resistance is increased in plants that overexpress *ARR22* (Kang et al., 2013). *A. thaliana* has a *MYB2* gene, which is activated by the ABA, which suppresses the *IPT* genes and lowers the level of cytokinin (Guo and Gan, 2011). In turn, this reduces the output of the AHK/AHP/ARR signalling cascade that aids the plants adaptation to drought and osmotic stress.

The interaction between SnRK2s, RRAs, and RRBs is another connection. The RRBs *ARR1*, *ARR11*, and *ARR12* physically engage with SnRK2s in non-stress situations, repressing their kinase activity and shutting off the drought response pathway. Furthermore, in drought-stressed plants, SnRK2s phosphorylate the *RRA ARR5*, inhibiting cytokinin signaling and limiting plant growth. These interactions demonstrate cytokinin regulates growth-trade-offs is well understood.

## Interactions of cytokinin with other phytohormones under abiotic stresses

Plant responses to abiotic stress conditions are mostly based on interactions among hormone signals. Cytokinin participates in a complex signal network with other phytohormone signaling pathways rather than playing a separate regulatory function. Cytokinin does not have a regulatory function that is independent of other phytohormone signaling pathways; rather, it acts within a complex signal network that includes several pathways (Li et al., 2016). Furthermore, coordinating tissue expansion in response to environmental changes requires the interaction of other phytohormone. As a result, the plant is able to respond rapidly to its changing environment due to a network of tightly interlinked signaling systems.

Abscisic acid (ABA) regulates one of the earliest plant drought responses, stomata closure, which controls the trade-off between CO_2_ intake and water loss via transpiration (Sah et al., 2016; Vishwakarma et al., 2017). Although ABA strongly interacts with cytokinins, it also regulates mid- and long-term plant responses to abiotic stress, including regulation of plant architecture. Accumulation of stress-induced ABA in turn downregulates cytokinin production by way of the MYB2 transcription factor (TF), alleviating the repression on multistep phosphorelay (MSP) and activating genes that are ABA- and stress-inducible (Li et al., 2016). Through the downregulation of shoot growth and the acceleration of root development, ABA-mediated suppression of cytokinin signaling starts the process of redesigning the plant body. This enables the plant to increase water intake from deeper soil layers while minimizing water loss (Li et al., 2016). Accordingly, ABA hypersensitivity and increased drought resistance are seen in MSP signaling mutants, such as those with defects in the cytokinin sensors AHK2, AHK3, and AHK4 and type-B ARRs ARR1, ARR10, and ARR16 (Tran et al., 2007; Tran et al., 2010; Nguyen et al., 2016). It has been demonstrated that ABA and drought may both downregulate the expression of *ARR1*, *ARR10*, and *ARR12* (Nguyen et al., 2016). According to Takatsuka and Umeda (2019), ABA also inhibits *ARR2* but not *AHK3* or *AHK4* and there may be a function for ABA in the regulation of AHP2’s nucleocytoplasmic partitioning (Marchadier and Hetherington, 2014). Tran et al. (2007) found that the osmosensor AHK1 is not a negative regulator of the ABA-mediated stress response, but rather a positive regulator. This suggests that there may be some specificity at the level of signals that start the MSP-regulated (drought) stress response (Hai et al., 2020).

There are two ways in which ABA interferes with MSP activity: ABA-controlled downregulation of the generation of cytokines and the interaction between ABA signaling components and MSP. ABA-activated ABI4 binds promoters and downregulates *ARR6*, *ARR7*, and *ARR15*; arr4, arr6, arr7, and arr15 mutant lines are hypersensitive to ABA (Jeon et al., 2010; Wang et al., 2011). ARR5, a type-A ARR and negative regulator of MSP signaling, has numerous Ser residues that are phosphorylated by SnRK2.2, SnRK2.3, and SnRK2.6. By inhibiting cytokinin signaling, this results in stability of the ARR5 protein, which improves ABA responsiveness and drought tolerance.

Dautel et al. (2016) postulated an AHK2/AHK3-dependent phosphorylation of Thr6 and Tyr19 of KIN10, one of the two subunits of SnRK1, acting under energy stress in their phosphoproteomic analysis (Baena-González and Sheen, 2008). According to KIN10-based global gene regulation (Radchuk et al., 2006; Baena-González et al., 2007), SnRK1 down-regulation has previously been linked to cytokinin and auxin signaling. However, ethylene signaling was found to be negatively regulated by SnRK1 phosphorylation-mediated inactivation of EIN3 (Kim et al., 2017), leading to a growth. There is a bidirectional negative link between ABA and cytokinin levels/signaling. ABA insensitivity in seed germination was caused by the overexpression of cytokinin production via the upregulation of AtIPT8 (Wang et al., 2011). In the process of seed germination, ABA insensitivity was caused by an increased cytokinin production brought about by an overexpression of *AtIPT8*. Additionally, ABA was unable to inhibit the expression of the type-A ARRs ARR4, ARR5, and ARR6 that physically interact with ABI5 and reduce *ABI5* levels when endogenous cytokinin levels are increased (Wang et al., 2011). The cytokinin-responsive type-B ARRs ARR1, ARR11, and ARR12 that physically engage with SnRK2s and suppress the kinase activity of SnRK2.6 are most likely the cause of the decreased sensitivity to ABA under high endogenous cytokinin levels. The cytokinin-dependent control of ABA signaling may be regulated at the transcriptional level by ARR10, which was shown to bind the promoters of multiple ABA signaling genes (Zubo et al., 2017).

Cytokinins suppress expression of the Arabidopsis HIGH-AFFINITY K + TRANSPORTER 1; 1 (AtHKT1; 1), which is responsible for removing sodium ions from root xylem, in response to salt stress through ARR1 and ARR12. This transporter is responsible for removing sodium ions. Additionally, it was shown that cytokinins controlled the type A response regulator ARR5’s expression in response to salt stress mostly *via* ARR1 and ARR12, demonstrating the role of specific MSP components in the roots in regulating sodium accumulation in the shoots (Mason et al., 2010).

The hormonal network underpinning the intricacy of plant responses to stress is also influenced by the ethylene (ET) pathway. ET has been investigated in the contexts of development and stress (Vanstraelen and Benková, 2012; Beguerisse-Díaz et al., 2013; Zhai et al., 2013), and it has most recently been shown to play a negative regulatory role in cold tolerance (Shi et al., 2012). Interestingly, cold stimulates the expression of *ARR5*, *ARR6*, *ARR7*, and *ARR15* in a manner similar to dehydration, most likely to inhibit cytokinin signal transduction and growth (Jeon et al., 2010; Kang et al., 2012). According to the findings of Shi et al. (2012), ethylene biosynthesis and signaling adversely affects the cold stress response in Arabidopsis. This is accomplished via the repression of cold-inducible *C-REPEAT BINDING FACTORS* (*CBFs*) (*CBF1*, *CBF2*, and *CBF3* genes), and the type-A ARR genes *ARR5*, *ARR7*, and *ARR15*. This ethylene-induced suppression was expected to be mediated by direct binding of EIN3 to the promoters of type-A ARRs, so possibly suggesting another mechanistic connection between classical ethylene signaling and MSP during plant desiccation.

Despite the fact that ET disrupts the cytokinin signaling pathway’s output, the pathway itself is also influenced by cytokinin. In fact, cytokinin is responsible for the stabilization of the enzymes 1-aminocyclopropane-1-carboxylate synthase 5 (ACS5) and ACS9 (Chae et al., 2003; Hansen et al., 2009), which are responsible for the conversion of S-adenosyl-methionine to 1-aminocyclopropane-1-carboxylic acid. This stability might result in an accumulation of ET, which would then have the potential to influence plant development processes such as root expansion (RůžiČka et al., 2007). According to Lehotai et al. (2012), the activation of both cytokinin and ET signaling in response to selenite-induced stress by means of the ARR5 and ACS8 markers and decrease in the levels of auxin suggests that the hormonal regulatory network that underlies stress responses is more complex than previously thought. Interestingly, there are tissue-specific characteristics in the cytokinin-ET and cytokinin-ABA interactions. Contrary to ET, which accumulates mostly in roots in response to high CK levels, CK treatments have been shown to enhance the accumulation of ABA in shoots but not in roots (Žd’árská et al., 2013).

## Priming as a strategy to develop abiotic stress tolerance

Cytokinin has been shown in the literature to be used as a priming agent to activate plant immune for biotic stress responses and biotrophic. Priming technology, on the other hand, is not widely used to protect plants from the negative effects of abiotic stressors or to prepare them to better withstand them. Moreover, it has been shown that priming the stress response pathways would be advantageous for the plant since it enables quicker and more robust responses with little energy expenditure. Although priming with several plant growth regulators (PGR) has been shown to be beneficial, evidence on employing cytokinins as priming agents is restricted to few experiments using kinetin or 6-benzylaminopurine (BAP). BAP has long been one of the cytokinins that is most often given to plants exogenously to dealyed senescence and decrease the impact of stress. Exogenous cytokinin treatment may reduce abiotic stressors on agricultural plants, resulting in enhanced growth, development, and yield. Similarly, cytokinin treatment lowers plant salinity stress (Ha et al., 2012) and promotes starch accumulation in salt-stressed rice plants (Javid et al., 2011).

Abiotic stress has been reduced in a variety of crop species by seed priming with cytokinins or a combination of cytokinins and other plant hormones. It is possible that genes associated to cytokinin play a significant role in the regulation of regeneration once a stress has been removed. Priming with cytokinins improves the production of chlorophyll (Chl) and the accumulation of biomass in plants. Additionally, it increases the photosynthetic rate, promotes membrane integrity, and keeps a stable ionic level. Wheat seeds primed with kinetin at concentrations of 100 mg L^−1^, 150 mg L^−1^, and 200 mg L^−1^ were shown to have improved germination and tolerance to salt. This was accomplished by lowering ABA concentrations and raising IAAs concentrations (Iqbal et al., 2006). Similar findings were made by Mangena (2020), who claimed that priming soybean seeds with cytokinins (Benzyl adenine; 4.87 mg L^−1^) improved soybean root biomass, flowering, and fruiting under drought stress. *Arachis hypogaea* L. aged groundnut seeds were primed with cytokinins (150 ppm), which improved antioxidant enzyme activities and reduced oxidative damage to improve germination and seedling indices (Sepehri et al., 2016). In addition, the mode of action of these PGRs in enhancing seed and plant fitness through priming has not been investigated. Moreover, it has been reported that exogenous application of cytokinins reduces ABA-induced stomatal closure because this PGR, which are important for stomatal movement, are involved (Tanaka et al., 2006). However, the effects of seed priming with cytokinins on stomatal movement remain unknown.

## Genetic engineering of cytokinin for improving or redesigning plant abiotic stress tolerance

Crop yield and production are threatened by abiotic factors such as severe temperatures, nutrient deficiency, low water levels, high salt concentrations and excessive light. Plants cytokinin mediated stress responses are highly dependent on the phytohormone concentrations (O’Brien and Benkova, 2013). Moreover, plants get acclimatized to stress as a result of both constitutive decrease and overproduction of cytokinins. As a result, precise manipulation will lead to altering its concentrations to achieve desired results (summarized in Table 1) (Rivero et al., 2007; Werner et al., 2010; Nishiyama et al., 2011; Ha et al., 2012). *A. thaliana* the model plant, has been the subject of the most extensive study on cytokinin-mediated stress responses till date (Ha et al., 2012). The most common method for lowering cytokinin levels is to change the expression of the *CKX* or *IPT* genes. Subsequently, the overexpression of *CKX* genes, as well as the disruption of *IPT* genes, will result in a reduce cytokinin levels. Furthermore, plants with cytokinin deficiency show bushy root growth, diminished apical dominance, and stunted shoot developmental phenotype. Nishiyama et al. (2011) used gain and loss-of-function mutants to show that the Arabidopsis cytokinin-overexpressing plants (*35S*:*CKX1*-*35S*:*CKX4*) and *ipt1, 3, 5, 7* quadruple mutant were more salt and droughts -tolerant than WT plants. Furthermore, root growth assays and intracellular electrolyte leakage measurements suggested that cytokinin deficient plants were more resistant to salinity stress owing to increased primary root development and more tolerant to drought because of improved cell membrane integrity (Nishiyama et al., 2011). Additionally, the reduction in cytokinin levels shown in *AtCKX*-overexpressing Arabidopsis transgenic plants had a major influence on the growth and development of several tissues, including roots and shoots, reproductive organs, floral, and vascular development (Werner et al., 2003). Root-specific expression of *CKX* in *N. tabacum* using the *W6*:*CKX1* construct (expression of *CKX1* driven by a *WRKY6* promoter) and in *A. thaliana* using the *P10*:*CKX3* construct (expression of *CKX3* driven by a *PYK10* promoter) revealed an enlargement of the root system architecture (RSA) in the transgenic lines, which showed similarity to the root feature of plants grafted between *35S*:*CKX1* or *35S*:*CKX3* (Werner et al., 2010). Furthermore, the transgenic plants accumulated more minerals, such as calcium, phosphate, molybdenum, and magnesium when compared with the WT (Werner et al., 2010). These data collectively support that the root development improved plants tolerance to water stress and nutrient deficiency.

Constitutive overexpression of cytokinin gives rise to severe anomalies in biological processes such as organogenesis, cell division, meristematic activities, and gametophyte development (Kieber, 2002). Because of this, organ-specific and stress-inducible cytokinin synthesis is thought to be more desirable. Gain-of-function studies, for example, showed that using stress-inducible promoters alternative to constitutive promoters might prevent growth abnormalities associated with endogenous cytokinin overexpression, such as dwarf and limited root growth phenotypes, results in improved control of cytokinin biosynthesis (Xing et al., 2009; Peleg and Blumwald, 2011). Several promoters, such as *HSP* (*heat shock protein*), *PSARK* (*senescence-associated receptor-like kinase*), *PSAG12* (*senescence-associated genes12*), and *rd29A* (*response to dehydration 29A*), have been successfully used to drive conditional expression of the *Agrobacterium tumefaciens* mediated *IPT* gene in *A. thaliana* (Zhang et al., 2000), tobacco (*N. tabacum*) (Rivero et al., 2007; Rivero et al., 2010), creeping bentgrass (*Agrostis stolonifera*) (Merewitz et al., 2010), rice (*O. sativa*) (Peleg et al., 2011), peanut (*Arachis hypogaea*) (Qin et al., 2011), cotton (*Gossypium hirsutum*) (Kuppu et al., 2013), and cassava (*Manihot esculenta*) (Zhang P. et al., 2010), to increase tolerance to a variety of stresses, including waterlogging and drought (Figure 2). Transgenic plants with increased cytokinin exhibited better adaptive responses to numerous stresses with an improvement in photosynthesis capacity, transpiration rate, intracellular water content, and delayed leaf senescence, all of which shows the potential to be useful and economical in agriculture.

The promoter *PSAG12* deriving the expression of the *IPT* gene significantly delayed the onset of leaf senescence but resulted in an unexpected change in source-sink relationships, nitrogen (N) mobilization, reproduction and growth in response to water stress were also reported (Jordi et al., 2000). Thus, an alternate promoter, *PSARK*, has been frequently employed to overcome such a problem, since this promoter may activate *IPT* expression prior to the onset of leaf senescence (Rivero et al., 2007; Reguera et al., 2013). Similarly, *A. thaliana* stress-induced *rd29A* overexpressed the *IPT* gene to confer salinity stress tolerance in *N. tabacum* (Qiu et al., 2012). Salt tolerance in transgenic *G. hirsutum* was improved by overexpressing the *A. tumefaciens IPT* gene using the *Ghcysp* (*G. hirsutum* cysteine proteinase) promoter, which is from the same family of cysteine endopeptidase genes as *SAG12* (Liu et al., 2012). Furthermore, when drought stress occurs during the vegetative stage of the *G. hirsutum* plant, this strategy proved efficient in enhancing plant performance, but drought stress after the flowering stage failed to provide a yield advantage (Zhu et al., 2018). Early flowering and a later heading date were caused by *PSAG39*:*IPT* expression in *O. sativa*. Under drought conditions, this was expected to assist plants to deal with modest water restrictions and increase grain yields (Zou et al., 2007; Liu et al., 2010). Additionally, increased *IPT* expression assisted the plants survival ability under stressful events and at the recovery stage under waterlogging and submerging situations (Huynh et al., 2005).

Heavy metal stress (HMs) has a negative impact on plant metabolic processes, particularly when zinc concentrations are elevated (Gill, 2014). When compared to WT, *PSAG12*:*IPT* transgenic *N. tabacum* displayed stronger protection against high zinc contamination by reducing transpiration rates and net photosynthetic while retaining free amino acids synthesis, which is suggestive of appropriate nitrogen (N) metabolism (Pavlíková et al., 2014). Furthermore, a lack of nutrients, particularly important minerals like N, may cause massive self-destructive processes within plant cells. *N. tabacum* transformed with the *PSARK*::*IPT* construct might aid in the inhibition of ROS (reactive oxygen species) formation and prevent the detrimental effects on plants induced by decreasing the N concentration (Rubio-Wilhelmi et al., 2011). Subsequently, another study employed the P*SAG12*:*IPT* construct to produce transgenic *A. stolonifera* that improved plant survival in the face of N or phosphate (P) deprivation (Zhang Y. et al., 2010).

Overexpression of *A. tumefaciens IPT* gene to increase endogenous cytokinins level as a countermeasure against adversarial temperature has also been implicated in many species, such as generating low temperature-tolerant sugarcane (*Saccharum* spp.) and cold-resistant tall fescue (*Festuca arundinacea*) using the Arabidopsis *COR15a* (cold-regulated gene15a) promoter and the maize ubiquitin promoter, respectively (Hu et al., 2005; Belintani et al., 2012). In response to heat stress, an effort was made on *A. stolonifera* utilizing HSP and PSAG12 promoters to overexpress the *IPT* gene from *A. tumefaciens* (Xing et al., 2009; Xu et al., 2009). Furthermore, Xing et al. (2009) have also established that *SAG12*-*ipt*- and *HSP18*-*ipt* bearing transgenic *A. stolonifera* exhibited significantly longer leaf life-span when compared to WT when subjected to dark and heat treatment, respectively. Another *A. thaliana* SAG family promoter, *SAG13*, may induce *IPT* expression in all mature leaves before senescence, similar to PSARK expression pattern, but with a more severe altered source-sink relationship (Swartzberg et al., 2006). Under salt stress, a modified strategy of employing root-specific cytokinin overproduction under the direction of a constitutive promoter might help *Solanum lycopersicum* (tomato) plants increase plant growth and yield (Ghanem et al., 2011). In salt-treated *S. lycopersicum* plants, root-to-shoot cytokinin transport was significantly boosted, resulting in better ion homeostasis, vegetative growth, delayed leaf senescence (in plants with root-specific *HSP70*:*IPT* expression), and increased fruit yield (Ghanem et al., 2011). Thus, this research proposed a unique effective technique to reduce salt-induced agricultural yield constraints.

Transiently increasing the cytokinin level *via* the crucial distance between the gene and its promoter is another application of the genetic engineering method. By utilizing the constitutive 35S promoter the *A. tumefaciens IPT* gene was fused to the downstream of other genes, like *AtGolS2* (Arabidopsis galactinol synthase) or *AOC* (*Bruguiera sexangula* allene oxide cyclase), which were involved in cold and salt stress tolerance, respectively (Guo et al., 2010). Subsequently, *A. thaliana* transgenic plants carrying the *pVKH35S*-*AOC*-*ipt* and *pVKH35S*-*AtGolS2*-*ipt* genes were able to achieve a small rise in cytokinin levels, resulting in improved plant development, higher chlorophyll production, and longer flowering (Guo et al., 2010). Another method of transiently increasing cytokinin activity is to modify the expression of O-glycosyltransferase moderately. In response to the successful isolation of the *ZOG1* (*Zeatin O-glucosyltransferase*) gene from the *Phaseolus lunatus* plant, which codes for the ZOG protein, transgenic *N. tabacum* expressing *35S*:*ZOG1* and *SAG12*:*ZOG1* transgenes were developed (Martin et al., 1999; Marie et al., 2008). Therefore, the stress-induced elevation in calcium levels aided the *SAG12*:*ZOG1*-transformed plants in establishing growth more quickly than the WT plants at the post-drought recovery stage, as compared to the WT plants. In contrast, transgenic plants that had the *35S*:*ZOG1* construct had a slower recovery rate, which suggests that having more cytokinin in the plant before a long and severe drought period could have a negative effect (Marie et al., 2008).

Conditionally or locally boosted cytokinin synthesis has been shown to improve plant growth and yield in *Brassica napus* (canola) and *A. stolonifera* utilizing various promoter and *IPT* gene combinations (Kant et al., 2015; Xu et al., 2016). In the field, yields of IPT transgenic *B. napus* were higher in both stressed and non-stressed conditions (Kant et al., 2015). The information that cytokinin is a negative regulator of elongation development of the main root and root branching has been used to develop another engineering strategy to increase tolerance to drought in plants (Werner et al., 2003). *A. thaliana*, *N. tabacum* and *Hordeum vulgare* roots had lowered cytokinin levels when *CKX* genes were only expressed in the roots. This led to a larger root system with mostly unaltered shoot growth and development (Werner et al., 2010; Macková et al., 2013; Ramireddy et al., 2018). A greater survival rate of *CKX* transgenic *N. tabacum* plants under drought stress in an intermixed planting revealed that these plants were more effective in competing for limited water resources than WT tobacco plants (Werner et al., 2010). Increased cytokinin degradation in the roots of transgenic *H. vulgare* (barley) resulted in a reduced stress response to long-term drought conditions which includes increased stomatal conductance and CO_2_ assimilation rates, decreased activation of critical ABA metabolism genes, and decreased build-up of ABA (Ramireddy et al., 2018). While large soil volume explored by *CKX* transgenic plants has been linked to some of these favourable benefits, other mechanisms, such as interplay between the cytokinin and ABA signalling pathways, may also be responsible for the altered response to drought stress in these plants (Vojta et al., 2016; Ramireddy et al., 2018).

Cytokinin related gene applications in genetic engineering have shown considerable promise for stress tolerance, leading to sustainable agriculture, however, they are primarily overexpressed research. Therefore, genetic engineering and breeding strategies leads to increase abiotic stress resistance by manipulating these genes. Although these molecular players have been extensively examined in non-crop plants such as *A. thaliana* and *N. tabacum*, they have yet to be investigated in agronomically important crops. Thus, the mechanism governing cytokinin signaling in economically significant crops may be an intriguing topic to investigate for abiotic stress improvement. Novel technology breakthroughs in the previous decade have highlighted the potential of *de novo* domestication of wild plants as a realistic approach for developing abiotic stress-tolerant crops while ensuring food safety and security. Several biotechnological strategies are being proposed to get a better knowledge of the cytokinin-related gene and various phytohormonal pathways involved in plant responses to abiotic stress. In order to generate stress-tolerant crops, new generation tools are now accessible that enable precise genome editing in specific genes. Genome editing is an excellent approach for speeding up the development of enhancing tolerance to abiotic stresses. However, there are only few studies that describe the use of CRISPR and cytokinin-related genes to enhance abiotic tolerance in commercially significant crops (Table 2) (Ogata et al., 2020; Wang et al., 2022). Clustered regularly interspaced short palindromic repeats (CRISPRs) and CRISPR associated (Cas) proteins, or CRISPR/Cas, when integrated with *de-novo* domestication becomes an ideal strategy for modifying plant genome that has a potential to be one of the most promising possibilities to enhance stress tolerance.

**TABLE 2:** A list of CK signaling genes involved in the development of abiotic stress-tolerant plants.

S. No.	Gene	Response to stress	Host plant	Genetic engineering approach	References
1	*ARR1*	↑Heat tolerance	*Arabidopsis thaliana*	Constitutive overexpression	Karunadasa et al. (2022)
2	*TaIPT8*	↑Drought tolerance	Wheat (*Triticum aestivum*)	CRISPR/Cas9-based gene editing and constitutive overexpression	Wang et al. (2022)
3	*IPT*	↑Salt tolerance	*Nicotiana tabacum*	Stress-inducible senescence overexpression	Avni et al. (2020)
4	*OsERA1*	↑Drought tolerance	Rice (*Oryza sativa*)	CRISPR/Cas9	Ogata et al. (2020)
5	*IPT*	↑Drought tolerance	Creeping bentgrass (*Agrostis stolonifera*)	Stress-inducible overexpression	Xu et al. (2017)
6	*CKX1*	↑Drought tolerance	Barley (*Hordeum vulgare*)	Constitutive overexpression	Pospíšilová et al. (2016)
7	*CKX1*	↑Drought tolerance	*N. tabacum*	Constitutive overexpression	Lubovská et al. (2014)
8	*IPT*	↑Zinc tolerance, ↓leaf senescence	*N. tabacum*	Senescence-inducible overexpression	Pavlíková et al. (2014)
9	*AHP2, AHP3, AHP5*	↑Drought tolerance	*A. thaliana*	Knockout	Nishiyama et al. (2013)
10	*ARR22*	↑Drought, ↑cold tolerance	*A. thaliana*	Constitutive overexpression	Kang et al. (2013)
11	*IPT*	↑Drought tolerance, ↓leaf senescence	Cotton (*Gossypium hirsutum*)	Senescence-inducible overexpression	Kuppu et al. (2013)
12	*IPT*	↑Cold tolerance, ↓leaf senescence	*Saccharum* spp.	Stress-inducible overexpression	Belintani et al. (2012)
13	*IPT*	↑Salt tolerance, ↓leaf senescence	*N. tabacum*	Stress-inducible overexpression	Qiu et al. (2012)
14	*IPT*	↑Salt tolerance, ↓leaf senescence	Cotton (*G. hirsutum*)	Senescence-inducible overexpression	Liu et al. (2012)
15	*AHK2, AHK3*	↑Drought, ↑cold, ↑salt tolerance	*A. thaliana*	Knockout	Kang et al. (2012)
16	*CKX1, CKX2, CKX3, CKX4*	↑Drought, ↑salt tolerance	*A. thaliana*	Constitutive overexpression	Nishiyama et al. (2011)
17	*IPT1, 3, 5, 7*	↑Drought, ↑salt tolerance	*A. thaliana*	Knockout	Nishiyama et al. (2011)

↑: Increase, ↓: Decrease.

## Future prospects

There is mounting evidence that cytokinin plays a number of roles in plant responses to various stress. Stress-related cytokinin signaling pathways and several genes that encode cytokinin metabolism enzymes have been identified as functionally significant, although little is known about their downstream components. Remarkably, the majority of the same components engaged in cytokinin regulated development are also implicated in the stress response. This suggests that there has been no distinct evolution of stress response modules, but rather the response to stress is intricately associated with the control of development. In this regard, a better understanding of cytokinins interactions with known stress response pathways would improve our understanding of the hormone’s function in regulating growth-defense trade-offs. To get a better understanding of the downstream events of the cytokinin signaling pathway and to identify linkages to traditional stress response pathways, refined genetic techniques and system analysis will be critical.

Many of the cytokinin responsive genes are engaged in signaling, metabolic, and transport systems that affect plant growth and development, and next-generation technologies have revealed insights into global transcriptome alterations in connection to cytokinin responsive genes (cytokinin response factors (CRFs), *CKXs, ARR1, ARR10,* and *ARR12*) (Shi et al., 2013; Abdelrahman et al., 2021). At the transcriptome and proteome levels, genome-wide investigations may reveal interaction protein–protein networks that regulates biological development processes in growing crop plants. Global insights into molecular mechanisms and genes involved in abiotic stress tolerance are viable targets for the development of novel strategies for crop improvements. Furthermore, many studies on the influence of cytokinins on stress are conducted in controlled conditions, suggesting that cytokinins are stress modulators that function through a growth-defense trade-off (Cortleven et al., 2019). Influences of cytokinins on genotype–environment interactions are still poorly understood in natural and/or in-field agricultural settings, and future studies should focus more rigorously on testing cytokinin stress modulation in natural environments for agricultural ecosystem management, especially in the context of climate change. Understanding the functions of cytokinin, a key growth-regulating hormone in stress defense is particularly vital for understanding the influence of a changing environment on plant development and ensuring the sustainability of food supply.

## Concluding remarks

The significance of cytokinins in the regulation of key developmental processes has become more apparent in recent years, providing new insights. While significant progress has been achieved, the true challenge remains in deciphering the molecular mechanisms by which cytokinins govern these developmental processes. In general, cytokinin signaling and metabolism are important for abiotic stress tolerance, and manipulating genes in the signaling pathway in major crops might be advantageous for long-term agricultural sustainability. Furthermore, the growing amount of molecular data adds to our understanding of cytokinin interplay in its developmental aspects while also adding a new degree of complexity. In addition, there are several crosstalk pathways with other plant hormones that aids to the cytokinin large pleiotropy in stress-induced growth regulation.

Furthermore, the genetic mechanism behind abiotic stress has been unravelled with the recent advancement in genomics and transcriptomics technologies. Stress tolerance genes in CWRs and other cultivated crops may be mapped using transcriptome profiling, a powerful tool. Because of recent developments in next-generation sequencing (NGS) technology, it is now possible to create high-quality pangenomes for a wide range of crops, giving researchers a full picture of genetic diversity within each species as well as the total gene pool for each specific crop. It is now feasible to implement next-generation breeding effectively for a complex trait like abiotic stress tolerance by combining *de novo* domestication with genome editing tools like CRISPR/Cas system.
